The article "Novel role of miR-133a-3p in repressing gastric cancer growth and metastasis via blocking autophagy-mediated glutaminolysis" was retracted in 2024. Reasons: duplicated images; overlap with earlier publications; unreliable data; concerns about the data.

# Novel role of miR-133a-3p in repressing gastric cancer growth and metastasis via blocking autophagy-mediated glutaminolysis

**DOI:** 10.1186/s13046-018-0993-y

**Published:** 2018-12-20

**Authors:** Xing Zhang, Zheng Li, Zhe Xuan, Penghui Xu, Weizhi Wang, Zheng Chen, Sen Wang, Guangli Sun, Jianghao Xu, Zekuan Xu

**Affiliations:** 1 Department of General Surgery, The First Affiliated Hospital of Nanjing Medical University, No.300, Guangzhou road, Nanjing, Jiangsu province China; 2 Department of Surgical Oncology, University of Miami, Miami, USA; 3 Collaborative Innovation Center For Cancer Personalized Medicine, Nanjing Medical University, Nanjing, 210029 Jiangsu Province China

**Keywords:** Gastric cancer, Autophagy, Glutaminolysis, miRNA, Organoid, GABARAPLI, PDX model

## Abstract

**Background:**

Autophagy plays a crucial role in sustaining the homeostasis in various malignant diseases. It has also been reported to promote tumor development in multiple cancers. Glutaminolysis instead of Warburg Effect produce adequate ATP and provide nitrogen and carbon to replenish the TCA cycle which has been discovered to be a new energy source for tumor cells recently. By means of degrading intracellular particles including amino acids, nucleotides, fatty acids, sugars and aged organisms, autophagy can recycle the aforementioned particles into bioenergetics and biosynthesis pathways, finally favoring tumor cells. MicroRNA is a kind of noncoding RNA that regulates the targeting gene expression mostly at post-transcription level. Among these miRNAs, microRNA-133a-3p is reported to be a tumor suppressor in numerous cancers.

**Methods:**

We characterized the down-regulated expression level of microRNA-133a-3p in gastric cancer via TCGA database. Subsequently, we verified the tumor suppressor role of microRNA-133a-3p in gastric cancer cells through a series biological function assay. We used immunofluorescence and transmission electron microscope to observe the negative effect of microRNA-133a-3p on autophagy and used dual-luciferase report assay to identify the candidate gene GABARAPL1 of microRNA-133A-3p.Then we used high performance liquid phase mass spectrometry and seahorse analysis to detect whether miR-133a-3p could block the glutaminolysis metabolism through autophagy. At last, we confirmed the tumor suppressor role of microRNA-133a-3p in vivo on PDX mice model.

**Results:**

We demonstrated that microRNA-133a-3p overexpression could block the activation of autophagy to ruin the abnormal glutaminolysis and further inhibit the growth and metastasis of gastric cancer cells. We successfully proved gastric cancer cells can replenish glutaminolysis via autophagy and microRNA-133a-3p could block aforementioned pathway by targeting core autophagy participants GABARAPL1 and ATG13.We then verified the negative function of microRNA-133a-3p on autophagy-mediated glutaminolysis both in PDX model and human gastric cancer organoid model.

**Conclusions:**

MicroRNA-133a-3p targets GABARAPL1 to block autophagy-mediated glutaminolysis, further repressing gastric cancer growth and metastasis.

**Electronic supplementary material:**

The online version of this article (10.1186/s13046-018-0993-y) contains supplementary material, which is available to authorized users.

## Background

Gastric cancer (GC for short), also recognized as stomach adenocarcinoma, is the fourth frequent cancer and the third leading cause of cancer-related deaths worldwide according to the GLOBOCAN database [1].Even with the development of the earlier diagnosis techniques and new therapeutic approaches, the 5-year overall survival remains poor, and less than 30% in most countries. GC is characterized as a highly heterogeneous solid tumor and featured with high autophagy, metabolic disturbance and hypoxia [2, 3]. Moreover, highly proliferative GC cells have to change their metabolism type to adjust to the severe micro-environment, eventually satisfying their needs for survival and metastasis [4].Therefore, it is an urgent need for us to understand the deeper molecular mechanism responsible for the GC progression and find new therapeutic targets or reliable diagnosis markers.

Autophagy plays a crucial role in sustaining the homeostasis of cells and various malignant diseases. For example, cancers may result from autophagy disfunction [5]. Autophagy has been reported to promote tumor development in multiple cancers. In addition to the role of autophagy on promoting resistance to chemotherapy [6], it is also known that autophagy may activate in hypoxic and energy-lacking conditions, which eases the stress on metabolism. By means of degrading intracellular particles including amino acids, nucleotides, fatty acids, sugars and aged organisms, autophagy can recycle the aforementioned particles into bioenergetics and biosynthesis pathways, finally enabling the survival of tumor cells [7]. Even with the sufficient energy, many tumor types demonstrate elevated autonomous basal autophagy. It was considered that the tumor metabolism mostly relied on glycolysis, also called Warburg Effect [8, 9], to meet its need for malignant behaviors. However, recent reports found that in certain tumor types, glycolysis itself could not entirely enable the survival of tumor cells under starvation, and glutaminolysis could fully rescue the survival of tumor cells instead. The pyruvate produced from the glycolysis has been finally transformed into lactate which does not directly replenish the tricarboxylic acid (TCA) cycle [10, 11]. Glutaminolysis enables glutamine transformed into glutamate by glutaminase (GLS), and then further being transformed into alpha-ketoglutarate (α-KG) by glutamate dehydrogenase(GDH) to produce adequate ATP and provide nitrogen and carbon to replenish the TCA cycle. Additionally, the glutaminolysis can help produce biosynthetic precursors which is necessary for cell growth and produce glutathione(GSH) to keep the ROS at a low level suitable for tumor cell proliferation [12–14]. Autophagy has been reported to mediate several types of metabolism to provide substrates for tumor survival including glycolysis and glutaminolysis [15–17]. However, the specific metabolic pathway and the regulation mechanism of glutaminolysis mediated by autophagy have not been explored in depth. Besides, there were reports proving that tumor metastasis mediated by epithelial–mesenchymal transition needs autophagy to sustain the viability of cancer cells [18–20]. Furthermore,PI3K/AKT/mTOR axis is publicly recognized to mediate the autophagy activation directly [21, 22] and promote EMT progression [23, 24] as well. However, the specific interaction between autophagy and EMT on GC metastasis remains to be explored in depth.

Autophagy-related genes (ATGs) are involved in multiple stages of autophagy which regulate the autophagosome formation [25]. Moreover, microRNAs (miRNAs) have been reported to regulate different ATGs to influence the autophagy [26–28].MicroRNAs (miRNAs) is a kind of noncoding RNA that functions mostly at the post-transcriptional regulation level and further regulates the targeting gene expression. They bind the 3′ untranslated region (3′-UTR) of their target mRNAs to work. Many studies have reported miRNAs play important roles in regulating carcinogenesis [29–31]. Some of them can affect proliferation, migration and invasion of tumor cells which make miRNAs themselves closely associated with clinical features including tumor stage, lymphatic invasion and patient survival. More and more studies discovered the diagnosis and prognosis value of certain miRNAs. Among these miRNAs, miR-133a-3p is reported to be a tumor suppressor in numerous cancer types including prostate cancer [32], gastric cancer [33], and bladder cancer [34] through multiple signaling pathways including PI3K/AKT/mTOR axis. However, the deeper regulation mechanism of miR-133a-3p in GC remains largely unknown. Recently, many people have reported miRNA could affect the activation of autophagy in stressful conditions such as starvation [35, 36].Therefore, we want to verify whether miR-133a-3p could break metabolic balance and EMT progression in GC by means of affecting the activation of autophagy, and ultimately limit GC cell proliferation, migration and invasion. We successfully found that GC cells use autophagy to recycle glutamine for glutaminolysis, and eventually ensure the survival of themselves and affect the EMT progression to promote metastasis. To summarize, miR-133a-3p acts as a crucial blocker on autophagy-derived pools of glutamine to inhibit GC development.

## Methods

### Tissue specimens

The tumor tissues and adjacent normal stomach mucosa tissues were collected from the GC patients who received radical gastrectomy at Department of Gastrointestinal Surgery, the First Affiliated Hospital of Nanjing Medical University from 2013 to 2017. All patients did not receive radiotherapy and chemotherapy before surgery. All the specimens were taken under the guidance of HIPAA protocol [37] and proved by the ethics committee. The TNM stage classification was followed TNM classification system of the International Union Against Cancer (7th edition) [38]. The disease free survival (DFS) is defined as the duration between the recurrence of GC and the primary GC. The overall survival(OS) is defined as the duration between the death of GC patients and the primary GC. We calculated the grouping of ROC curve according to the cut-off value of miR-133a-3p relative expression and the middle expression of miR-133a-3p.

### Cell culture and lentivirus transfection

The human GC cell lines BGC-823,SGC-7901,MGC-803,MKN-45,HGC-27,AGS and normal stomach mucosa epithelium cells GES-1 were all purchased from the Cell Center of Shanghai Institutes for Biological Sciences. AGS cells were cultured in F12K medium with the supplementation of 10% fetal bovine serum (Invitrogen), while the GC cells were all cultured in RPMI-1640 medium with the supplementation of 10% fetal bovine serum (Invitrogen). Moreover Antibiotics(1% streptomycin/penicillin, Gibco, USA) were added in the aforementioned culture system which were set at 37 °C in a moisture air under 5% CO2. We seeded 2 × 10^5^ BGC-823 and MKN-45 cells in 6-well plate overnight and then washed these cells with PBS for three times and these cells were finally both received overexpression lentivirus(LV-miR-133a-3p) and interference lentivirus (LV-miR-133a-3p IN) (MOI, 100 for BGC-823; 20 for MKN-45) by the supplementation of Polybrene (8 mg/ml). Subsequently we used RT-PCR to verify the transfection efficiency. The sequence we used for miR-133a-3p overexpression (5’ UUUGGUCCCCUUCAACCAGCUG 3′) and the sequence we used for miR-133a-3p-IN (5’ CAGCUGGUUGAAGGGGACCAAA 3′) were cloned into LV12-U6/luci05/puro vector (GenePharma, Shanghai, China). The LV12 empty lentiviral construct(LV-NC) served as a negative control and was taken to transfect BGC-823 and MKN-45 GC cells in the same approach. We successfully kept the stable clones of miR-133a-3p in GC cell lines by adding puromycin up to 5 μg/ml gradually (Sigma, Aldrich) until 5 days. Genepharma Biotech (Shanghai, China) constructed shRNA vectors targeting GLS (GLS siRNA).

### Reagents and antibodies

Hydroxychloroquine (HCQ), BPTES(H0915, SML0601) were purchased from Sigma-Aldrich (Shanghai, China). Regarding the primary antibodies used in the study, anti-GLS(ab93434), anti-ULK1(ab128859),anti-ATG5(ab108327), anti-GABARAPL1(ab86497), and anti-ATG13(ab214074) were purchased from Abcam (Cambridge, UK); Anti-GDH was purchased from Shybio (Shanghai, China); Anti-LC3A/B (12741), anti-Beclin-1 (3495), anti-SQSTM/p62(8025), anti-ATG7(2631),anti-mTOR (2983), anti-phospho-mTOR(5536,1230), anti-AKT(4685), anti-phospho-AKT(4060), anti-E-Cadherin (3195), anti-N-Cadherin(13116), anti-Slug(9585), anti-Snail(3879) and anti-TWSIT1(46072) were purchased from Cell Signaling Technology (Danvers, PA USA).

### Clonogenic assay and clonogenic survival assay

For clonogenic assay,we seeded LV-miR-133a-3p, LV-miR-133a-3p-IN and LV-miR-NC GC cells in 6-well plates (500 cells per well) for 2 weeks. For clonogenic survival assay, we seeded aforementioned cells in 6-well plates and cultured them with normal growth medium PRMI1640 with 10% fetal bovine serum. Subsequently we replaced the original culture medium with FBS-free RPMI1640 when GC cells were at 80% confluence in the well for 2 days. Furthermore, all the aforementioned cells in plates were fixed in 2 ml of methanol for 30 mins and stained with crystal violet for 20 mins.

### Quantitative real-time reverse transcription polymerase chain reaction(qRT-PCR)

Trizol Reagent(Invitrogen,15,596,018) were used to extract RNA from GC cell lines and tumor tissues. We used PrimeScript RT Master Mix Kit (TaKaRa, RR036A, Japan) to reverse-transcribe the mRNA and New Poly(A) Tailing Kit (ThermoFisher Scientific, China) to reverse-transcribed the miRNA both into cDNA. Subsequently we used Universal SYBR Green Master Mix (4,913,914,001, Roche, Shanghai, China) to perform polymerase chain reactions in order to amplify the cDNA to the same quantity level. We used 2^-△△CT^ analysis method to calculate the Ct value during the exponential amplification phase. Meanwhile, we used β-actin and RNU6–1 as the internal references for mRNA and miRNA respectively.

### Protein extraction and western blot assay

All proteins within cells and tissues were extracted by the iced lysis buffer(Cell Signaling Technology, Danvers, Massachusetts, U.S.) under the supplementation of a mixture of protease inhibitor(Calbiochem, Darmstadt, Germany). Subsequently, we used BCA assay Kit (Pierce, Rockford, IL) to determine the protein concentration of different samples and used the lysis buffer to adjust all the samples to the same concentration. Furthermore, equal quantity of protein extracts were added with 10% SDS–PAGE and were then boiled until denaturation.

For the western blot, we transferred the aforementioned protein extracts into nitrocellulose membranes. Subsequently we blocked the membranes with 0.05% Tween in TBST buffer, and then we used the specific primary antibody to incubate at 4 °C overnight. The membranes were washed in TBST for 10 mins for 3 times at room temperature on the next day. Furthermore, we used the second antibody targeting the primary antibody for 2 h at room temperature and also washed with the aforementioned protocol. Finally, we used chemiluminescence detection system to determine the bands.

### Transmission electron microscopy (TEM)

We fixed the MKN-45 and BGC-823 GC cells with 2.5% glutaraldehyde at 4 °C overnight. Subsequently, we used 1% OsO4 to continue to fix the cell samples. In the following step, we used ethanol and propylene oxide to dehydrate the cell samples. We cut samples into slide sections and stained them with 0.3% lead citrate before we finally took a JEM-1010 electron microscope (JEOL, Tokyo, Japan, 2500x or 8800x magnification) to detect the autophagosomes,

### ROS detection with DHE staining

The cells were washed with PBS buffer twice and then were stained with DHE (Sigma, D7008) (20 μmol/L) at 37 °C for 30 mins. Subsequently, we took fluorescence microscope to observe the red fluorescence to determine the ROS level.

### Dual-luciferase reporter assay

We cloned into pMIR-REPORT plasmid (H306, Obio Technology, Shanghai, China) with 3’UTRs containing wild-type or mutant miR-133a-3p response elements from GABARAPL1 and ATG13. We used Lipofectamine 3000 to transfect the reporter plasmid into GC cells. For the last step, we used DualLuciferase Reporter System Kit (E1910, Promega, USA) to indicate the Firefly and Renilla luciferase activity.

### 5-Ethynyl-2′-deoxyuridine (EdU) assay

We used EdU assay kit (RiboBio, China) to detect the DNA synthesis and cell proliferation. We seeded 10,000 treated GC cells into a 96-well plate overnignt. On the next day, we added Edu solution (25 μM) into the 96-well plates for 24 h.Subseuently we used 4% formalin to fix the GC cells at room temperature for 2 h. In the following step, we used 0.5% TritonX-100 to permeabilize the GC cells for 10 mins. We then added 1× Apollo reaction solution(200 μl) to stain the EdU for 30 mins and Hoechest33342 (200 μl) to stain the nuclei. Finally, we used Nikon microscope (Nikon, Japan) to observe the DNA synthesis and cell proliferation reflected by red and blue signals.

### The detection of oxygen consumption rate (OCR)

We used Seahorse Biosciences metabolism analyzer (XF24) to detect the oxygen consumption rate of GC cells. We seeded 2.5 × 10^4^ GC cells per well in the 24-well plates and we submitted them to metabolism assay after 24 h. Real-time OCR was measured every 15 mins for 3 h. We normalized the relative oxygen consumption rate to the 0-min time point.

### LC-MS detection for glutaminolysis products

We washed treated GC cells in the plates with PBS twice to wipe off the dead cells. In the next step, we add cell samples in 2 ml premixed 80% methanol solution under − 80 °C. Subsequently, we used 0.5 ml additional 80% methanol solution to re-extract the insoluble particles for 5 min on dry ice. Continuously, we combined supernatants which collected at each extraction to dry under N2 and reconstituted them in specific LC-MS testing water. After this task, we took reversed-phase ion-pairing chromatography coupled by negative mode electrospray ionization to a stand-alone Orbitrap mass spectrometer (Thermo Scientific) to detect the amino acids within the samples. It used solvent A (97:3 H2O/MeOH with 10 mM tributylamine, 15 mM acetic acid) and solvent B (100% MeOH) to detect from m/z 85–1000 at 1 Hz at 100,000 resolution with LC separation on a Synergy Hydro-RP column (100 mm × 2 mm, 2.5-μm particle size; Phenomenex). The concentration of several amino acids were finally determined with Maven software.

### CCK-8 assay

We used the Cell Counting Kit-8 assay (Dojindo Laboratories, Kumamoto, Japan) to determine the proliferation rate of GC cells. Firstly, we seeded 1000 cells into 96-well plates to observe for 7 days. Each day we added 10 ml CCK-8 solution to a new well at 37 °C for 2 h. Following this,we took automatic microplate reader (BioTek, Winooski, VT, USA) to measure at the absorbance at 450 nm to compare numbers on each day.

### Cell migration and invasion assay

The methods used for migration assay and invasion assay are almost the same. We put transwell assay inserts (Millipore, Billerica, MA, USA) in a well of 24-well plates. However,the difference is the membrane in the upper chamber of transwell assay in invasion assay is Matrigel-coated membrane(BD Biosciences) while the one in migration assay is only a normal membrane. In the experiment, firstly, we set 500ul serum-free RPMI1640 at bottom chamber. Following this, we seeded 10,000 cells in 200ul RPMI1640 with 10% FBS at upper chamber. After 24 h or 48 h, we used methanol to fix the cells within the membrane and stain them with crystal violet. Our final task is to observe these cells by microscope.

### Human gastric organoid model

We followed the previously reported method [39] to construct human gastric organoid model and investigate the regulation role of miR-133a-3p in a micro-environment similar to human condition. We transfected the organoids with LV-miR-133a-3p-IN,LV-miR-133a-3p and LV-NC, and used microscope to observe the growth of organoids on each day. We harvested the GC organoids from the Matrigel to be fixed in 70% ethanol and wrapped into paraffin sections to prepare for immunofluorescence staining.

### Immunofluorescence analysis of GC cells

We seeded 2000 GC cells in specially designed confocal dish cultured with RPMI1640 with 10% fetal bovine serum for one night. We used PBS to wash the plates twice and then fixed the GC cell with 4% formaldehyde solution for 30 mins at room temperature. Following this, we used PBS to wash plates twice again before we used 0.2% Triton X-100 to make GC cells more permeable.1% BSA was used to block the non-specific binding sites before we used primary antibody from different species to bind the specific location within GC cells or human gastric organoid at 4 °C. At last, we used second antibody Cy™ 3-Goat Anti-Rabbit IgG (Jackson, 1:100) to bind the primary antibody for 2 h and DAPI to stain nucleus for 15mins. At last, we used confocal microscope(Nikon, Japan) to observe the fluorescence signal.

### Immunohistochemical (IHC) analysis of tissue samples

We used 10% formalin to fix GC tissues and xenografted tissues and embedded them with paraffin. After the embedment, we cut GC tissues into slides and used primary body to specifically bind the respective targets overnight at 4 °C. On the next day, we used PBS to wash them twice and used HRP-Polymer-conjugated secondary antibody (Abcam, UK) to incubate tissues at room temperature for 1 h. Subsequently, we used 3,3-diaminobenzidine solution and hematoxylin to stain the samples. Lastly, we used microscope to observe the positive tumors and intensity of stained cells.

### Hematoxylin and eosin staining of tissue

Firstly, we used a microscope slide to rehydrate the tissue samples fixed in alcohol. Subsequently we agitated the slides for 30s in deionized water to hydrate the tissues. Subsequently, we put the slides into a bottle filled with hematoxylin and agitate for 30s and washed them in deionized water for 30s. After the previous steps, we used 1% eosin Y solution to stain the slide and rehydrated the sample with 95% alcohol and 100% alcohol. We took xylene to extract the alcohol continuously. In the last step, we covered the slides and used microscope to observe.

### Patient derived xenograft model(PDX model)

Firstly, we kept the tissues in iced RPMI1640 with 10% fetal bovine serum and cut them into 2*2*3 Mm^3^ and then used the fresh RPMI1640 to wash tissues twice. Before we finished residure procedures, we kept tissues in PRMI1640 with the supplementation with penicillin and streptomycin.NOD/SCID mice was chosen to be the first generation PDX mice that carried the patients’ tissues. We used 10% chloral hydrate(0.004 ml/g) to make mice into anesthetized condition. By sterile operation, we buried tumor tissues on the mice back subcutaneously with the supplementation of penicillin and streptomycin at the same time. The rest PDX generation mice were BLAB/c-nude mice. When each xenografted tumor tissue grew up to 1–2 cm^3^,we followed the same protocols to harvest the tissues and transplanted them into the next generation mice immediately for four times until the 4th BLAB/c-nude. We injected the recombinant lentivirus vectors or drugs into tumor tissues continuously from day 0 to day 20, and then harvested the tumor tissues to received further analysis at day 40.

### In vivo metastasis assay

Firefly luciferase gene was stably transduced into miR-133a-3p lentivirus vectors. We injected the vectors through tail vein of BALB/c nude mice. At the last step, we observed the bioluminescent signal after injecting 100 mg/kg of D-luciferin (Xenogen, Hopkinton, MA) into mice with an IVIS 100 Imaging System (Xenogen).

## Results

### Identification of the down-regulated expression profile of miR-133a-3p in GC tissues from TCGA database

To determine the expression pattern of miRNAs in GC tissues, we downloaded the up to date miRNAs-seq data that comprised 446 GC samples and 45 normal samples from the Cancer Genome Atlas (TCGA) datasets. We analyzed the variation of miRNA expression between GC and normal samples by volcano plots (Fig. 1a). In total, 319 differentially expressed miRNAs with fold-changes greater than 2.0 were validated, among which 96 miRNAs were downregulated and 223 miRNAs were upregulated. The cluster heat map presented the top 40 differentially expressed miRNAs according to the expression level (Fig. 1b). The top 10 downregulated and top 10 upregulated miRNAs were listed in the following figure (Fig. 1c). The miR-133a-3p (mature sequence of miR-133-1,2) was downregulated more than 3 folds combined with its most significant *P* value which attracted our attention and we also showed its expression pattern from TCGA miRNAs-seq (Fig. 1d). To further validate the expression profile of miRNAs from TCGA database, we performed qRT-PCR assay among 80 paired GC tissues and adjacent normal tissues from 80 patients and observed the consistent results with the database (Fig. 1e). Subsequently, we analyzed the clinical and pathological data of these 80 patients and we found the downregulation of miR-133a-3p is significantly correlated with the tumor size and lymphatic invasion of GC patients (Table 1). We plotted the overall survival(OS) and disease-free survival (DFS) curves by KaplaneMeier method according to the circNRIP1 expression level. Longer OS (median survival of 55 months vs 21 months; *P* = 0.0009, log-rank test; Fig. 1f) and DFS (median survival of 52 months vs 19 months;*P* = 0.0008, log-rank test; Fig. 1f) were observed in patients with high levels of circNRIP1 compared with those the low levels of circNRIP1.Thus, we attempted to understand the deep mechanism of the tumor suppressor role of miR-133a-3p.

**Fig. 1:** Identification of the down-regulated expression profile of miR-133a-3p in GC tissues from TCGA database. (**a**) 319 differentially expressed miRNAs according to TCGA miR-seq with fold-changes greater than 2.0 were showed by volcano plots. (**b**). The cluster heat map which demonstrates the top 40 differentially expressed miRNA. Rows represent circRNAs while columns represent tissues. (**c**). The top 10 downregulated and top 10 upregulated miRNAs were listed. (**d**). Expression pattern of miR-133a-3p from TCGA miR-seq. (**e**).qRT-PCR assay among 80 patients showed the consistent results with the database. (**f**). Overall survival(OS) and disease-free survival (DFS) curves were plotted by KaplaneMeier analysis according to the circNRIP1 expression level. All data are presented as mean ± SEM. *p < 0.05, **p < 0.01, ***p < 0.001

**Table 1:** Association between the expression level of miR-133a-3p or GAPARAPL1 and the clinical characteristics in GC patients

Parameters	Group	miR-133a-3p expression				GABARAPL1 expression			
		Cases	Low	High	*P*-value	Cases	Low	High	*P-value*
Gender	female male	24 56	13 27	11 29	0.6256	15 35	7 18	8 17	0.7576
Age at surgery	≥ 55 < 55	64 16	29 11	35 5	0.0935	7 43	5 20	2 23	0.2214
T grade	T1 + T2 T3 + T4	45 35	21 19	24 16	0.4990	24 26	14 11	10 15	0.2575
Lymphatic invasion	Negative(N0) Positiv(N1-N3)	23 57	7 33	16 24	0.0262*	20 30	12 13	8 17	0.2482
Tumor site	Cardiac Non-cardiac	30 50	16 24	14 26	0.6442	18 32	12 13	6 19	0.0771
Stage	I-II III-IV	41 39	18 22	23 17	0.2634	23 27	14 11	9 16	0.1560
Size(cm)	< 3 ≥ 3	37 43	13 27	24 162	0.0136*	21 29	14 11	7 18	0.0449*
Histology grade	Well-moderately Poorly-signet	25 55	15 25	10 30	0.2278 0.	17 33	10 15	7 18	0.3705

*P* < 0.05 represents statistical significance (Chi-square test)

### Restoration of miR-133a-3p expression inhibits proliferation,migration and invasion abilities of GC cell and organoid model

To better understand the biological function of miR-133a-3p on GC development, we determined its expression level among several GC cell lines. We verified the down-regulated expression level of miR-133a-3p in GC cell lines compared to the GES-1 cell (normal gastric mucosa epithelial cell).and chose the first highest BGC-823 GC cell line and the second highest MKN-45 cell line to investigate the downstream mechanism of miR-133a-3p in GC development (Fig. 2a). We transfected the MKN-45 and BGC-823 cells with miR-133a-3p mimics, inhibitor and NC(negative control). Transfection efficiency of miR-133 mimic and miR-133a-3p inhibitor in both cell lines were confirmed (Fig. 6c). Cell proliferation in miR-133a-3p transfected GC cells was analyzed by CCK-8 assay and Edu assay. Upregulation of miR-133a-3p in GC cells significantly reduced the proliferation rate(Fig. 2b) and DNA synthesis (Fig. 2c).

**Fig. 2:** Restoration of miR-133a-3p expression inhibits proliferation,migration and invasion abilities of GC cell and organoid model. (**a**). Expression levels of miR-133a-3p among several GC cell lines. (**b**). Proliferation rate was analyzed by CCK8 assay.miR-133a-3p overexpression suppressed the proliferation of GC cells while the miR-133a-3p-IN had the opposite effect. (**c**) DNA synthesis was analyzed by Edu assay.miR-133a-3p overexpression suppressed the DNA synthesis of GC cells while the miR-133a-3p-IN had the opposite effect, scale bar = 100 μm. (**d**). The clonogenicity of both miR-133a-3p mimic and inhibitor transfected cells were assessed. (**e**). Migration and Invasion abilities of GC cells were supprresed under miR-133a-3p mimics while the miR-133a-3p-IN had the opposite effect, scale bar = 200 μm. (**f**). We found that overexpression of miR-133a-3p could significantly block the growth of GC organoid, whereas miR-133a-3p knockdown could promote GC growth, scale bar = 50 μm. All data are presented as mean ± SEM. *p < 0.05, **p < 0.01, ***p < 0.001

It was observed the opposite effect of the miR-133a-3p inhibitors group compared with the negative control (Fig. 2b,c). Furthermore, the clonogenicity of both miR-133a-3p mimic and inhibitor transfected cells were assessed, and we found that miR-133a-3p overexpression significantly reduced the number and size of colonies inoculated after 14 days compared with NC group, while the miR-133a-3p inhibitors promoted the clonogenicity (Fig. 2d). Moreover, we analyzed the effect of ectopic miR-133a-3p expression on cellular migration and invasion potential of MKN-45 and BGC-823 cells. Upregulation of miR-133a-3p significantly suppressed the ability of GC cells to migrate through normal transwell membrane(Fig. 2e). In addition, overexpression of miR-133a-3p significantly inhibited GC cells invasion from entering matrigel-coated transwell membranes (Fig. 2e). The miR-133a-3p inhibitors transfected GC cells were observed the opposite outcome (Fig. 2e). At the very last,the 3D GC organoid model was further taken to investigate the biological role of miR-133a-3p on GC growth. And GC organoid model could highly phenocopy the tumor microenvironment in vivo. We found that overexpression of miR-133a-3p could significantly block the growth of GC organoid, whereas miR-133a-3p knockdown could promote GC growth (Fig. 2f). Collectively, these results suggested the tumor suppressor role of miR-133a-3p on gastric tumor development in the aspect of inhibiting proliferation and metastasis.

### Low level of miR-133a-3p is responsible for the induction of autophagy especially in starvation

Forwardly, we attempted to figure out the underlying molecular mechanism by which the miR-133a-3p induced inhibition on GC cell proliferation,invasion and migration. Autophagy has emerged as a critical regulator of the malignancy of cancer [40, 41]. During the starvation, autophagy recycles the captured components to sustain macromolecular synthesis, anaplerosis, and energy production for the survival and metastasis [42, 43] of tumor cells. We herein explored the effects of miR-133a-3p on autophagy. Overexpression of miR-133a-3p successfully blocks the serum deprivation-induced autophagy in MKN-45 and BGC-823 cells (Fig. 3a, b, c). Autophagosomes were evaluated in transfected GC cells by transmission electron microscopy (TEM), confocal laser scanning microscope (CLSM) and western blot. TEM results suggest a remarkable accumulation of autophagosomes in the cytoplasm of miR-133a-3p inhibitors transfected GC cells compared with miR-133a-3p mimics transfected cells under starvation (Fig. 3a). Autophagosome formation is a complex procedure. It is already discovered that ULK1, beclin-1,ATG 5 and ATG 7 are the major participants in autophagy initiation, vesicle nucleation and vesicle elongation respectively. We used western blot analysis to observe them and the classical hall marker SQSTM1(P62) and LC3 in GC cells. Decreased expression levels of autophagy markers can be observed in miR-133a-3p mimics transfected GC cells. And it was observed an opposite effect of miR-133a-3p inhibitors transfected GC cells (Fig. 3b). In addition, we observed that among multiple autophagy targets, the ULK1 and beclin-1 appeared to be the most up-regulated (Fig. 3b). Therefore, the conclusion could be arrived at that miR-133a-3p impact autophagy especially the initiation and vesicle nucleation stages. To further verify aforementioned results, we then established two GC cell lines that stably expresses an mRFP-GFP-LC3 fusion protein. MiR-133a-3p inhibitors transfected cells showed a stronger mRFP-GFP-LC3 signal compared with miR-133a-3p mimics and negative control transfected cells (Fig. 3c). To summary, these results suggest that the knockdown of miR-133a-3p could promote autophagy, especially in initiation and vesicle nucleation stages under starvation. Besides, considering the miR-133a-3p role on metastasis ability of GC cells and the positive interaction between autophagy and EMT [44, 45] were reported these years, we used western blot to determine the suppressor role of miR-133a-3p on EMT in MKN-45 and BGC-823 GC cells (Fig. 3d). The GC organoid model was further taken to demonstrated the negative function of miR-133a-3p on autophagy, EMT and proliferation. Finally, we observed the increased expression levels of proliferation marker Ki67 and autophagy marker LC3 as well as the decreased expression level of EMT marker E-cadherin by immunofluorescence in GC organoid models under miR-133a-3p inhibitors treatment compared with negative control(Fig. 3e). Thus, the suppressor role of miR-133a-3p on autophagy and EMT was proved by us.

**Fig. 3:** Low level of miR-133a-3p is responsible for the induction of autophagy especially in starvation**.** (**a**). We used TEM to observe a remarkable accumulation of autophagosomes in the cytoplasm of miR-133a-3p inhibitors transfected GC cells compared with miR-133a-3p mimics transfected cells under starvation. (**b**). Decreased expression levels of autophagy markers can be observed in miR-133a-3p mimics transfected GC cells. While miR-133a-3p inhibitors transfected cells can be observed an opposite effect. (**c**). MiR-133a-3p inhibitors transfected cells showed a higher mRFP-GFP-LC3 signal compared with miR-133a-3p mimics and negative control transfected cells, scale bar = 10 μm. (**d**). Increased trend of EMT was observed in miR-133a-3p IN transfected GC cells while the opposite trend of EMT was observed in miR-133a-3p mimics transfected GC cells compared with NC transfected GC cells by western blot. (**e**). We observed the increased expression levels of proliferation marker Ki67, EMT marker E-cadherin and autophagy marker LC3 by immunofluorescence in GC organoid models under miR-133a-3p inhibitors treatment compared with negative control, scale bar = 50 μm. All data are presented as mean ± SEM. *p < 0.05, **p < 0.01, ***p < 0.001

### Identification of GABARAPL1 as the target of miR-133a-3p which is responsible for the autophagy activation and mediating the proliferation and metastasis abilities of GC cells

To understand the mechanism of autophagy inhibition by miR-133a-3p in depth, we utilized several bioinformatic databases including Targetscan, miRanda and miRbase to cross analyze the potential autophagy-related target genes of miR-133a-3p. Thus we identified GABARAPL1 as a probable target of miR-133a-3p according to the high matching score (Fig. 4a). It was reported that GABARAP (ATG8) subfamily proteins served as scaffolding proteins by recruiting ULK1 and beclin-1 (complex) to the site of autophagosome nucleation and directly participant autophagy more efficiently than LC3 [46, 47]. Therefore the 3’-UTR (3′-untranslated region) of GABARAPL1 (GAU), the wide-type (GAU-WT) or mutant (GAU-MT) of putative miR-133a-3p binding sequence was respectively cloned into pmirGLO dual-luciferase reporter vector (Fig. 4b). The luciferase signal significantly decreased in MKN-45 and BGC-823 cells after co-transfection of miR-133a-3p mimics with GAU-WT for 48 h compared with negative control. On the contrary, the luciferase signal of GAU-MT did not change upon the inhibition of miR-133a-3p mimics (Fig. 4c). These results proved that miR-133a-3p targets the 3’-UTR of GABARAPL1 mRNA. Moreover, ULK1 is reported to be a member of a crucial autophagy-related complex and it is implicated in autophagosome formation by phosphorylating beclin-1.

**Fig. 4:** Identification of GABARAPL1 as the potential target of miR-133a-3p which is responsible for the autophagy activation and mediating the proliferation and metastasis abilities of GC cells. (**a**). Bioinfomatic predictions of targeting genes of miR-133a-3p; (**b**). Wild and mutant sequences of GABRAPL1 and ATG13; (**c**). The luciferase signal significantly decreased in MKN-45 and BGC-823 cells after co-transfection of miR-133a-3p mimics with GAU-WT (ATU-WT) for 48 h. On the contrary, the luciferase signal of GAU-MT (ATU-MT) did not change upon the inhibition of miR-133a-3p mimics. (**d**). Western blot demonstrated that either knocking down GABARAPL1 or using HCQ could reverse the promotor role of miR-133a-3p IN on autophagy and EMT; (**e**). We further detected the negative correlation between the expression of miR-133a-3p and GABARAPL1 by performing qRT-PCR among 50 gastric cancer tissues; (**f**).CCK8 assay showed that the positive role on GC proliferation rates of miR-133a-3p inhibitors was successfully reversed by GABARAPL1 siRNA and HCQ, scale bar = 200 μm. All data are presented as mean ± SEM. *p < 0.05, **p < 0.01, ***p < 0.001

Similarly, ATG13, an initiation promoter, was also identified as a potential target of miR-133a-3p (Fig. 4b). We constructed the 3’ UTR reporters of ATG13 containing the putative miR-133a-3p binding sites and the corresponding mutant constructs the downstream of the luciferase reporters. GC cells were co-transfected with various combinations of luciferase reporter vectors which were transfected with either empty luciferase vector, luciferase vector containing wild-type ATG13–3’UTR (ATU-WT), or luciferase vector containing mutant-type ATG13–3’UTR (ATU-MUT) and miR-133a-3p mimics. In cells transfected with the ATU-WT and the miR-133a-3p mimic, we observed a significant weakened luciferase signal compared to other groups (Fig. 4c). Aforementioned results indicated that miR-133a-3p might also directly interacts with the 3’-UTR of ATG13 to mediate its autophagy formation function besides GABARAPL1.

Furthermore, the expression of GABARAPL1 and ATG13 in MKN-45 and BGC-823 GC cells under starvation were determined (Fig. 4d). We detected that the expression level of GABARAPL1 and ATG13 were reduced in miR-133a-3p mimics transfected MKN-45 and BGC-823 cells, whereas the GABARAPL1 and ATG13 expression level increased in miR-133a-3p inhibitors transfected GC cells. These results demonstrated that the endogenous miR-133a-3p could target two key autophagy-associated genes, which are involved in autophagy induction and vesicle nucleation to inhibit autophagy in gastric cancer cells.

In the next step, we chose GABARAPL1 to investigate the downstream regulation mechanism of miR-133a-3p on GC development according to the higher complementarity between GABARAPL1 and miR-133a-3p compared to the ATG13 indicated by the dual-luciferase report assay. We further detected the negative correlation between the expression of miR-133a-3p and GABARAPL1 by performing qRT-PCR among 50 gastric cancer tissues (Fig. 4e,R^2^ = 0.2544,*P* < 0.05). In order to confirm the suppressor role on GC cells of miR-133a-3p which was mediated by autophagy via targeting GABARAPL1,we treated the miR-133a-3p inhibitors transfected GC cells with GABARAPL1 siRNA, hydroxychloroquine (HCQ,25 μm,an autophagy inhibition drug) respectively. We also transfected the GABARAPL1 overexpression plasmid into miR-133a-3p mimics GC cells. Next, we detected the proliferation and metastasis abilities of GC cells under aforementioned treatments by CCK8 assay, colony formation assay, Edu assay and transwell assay. We found the promotor role of miR-133a-3p inhibitors on GC malignant behaviors was successfully reversed by GABARAPL1 siRNA and HCQ including the proliferation rates (Fig. 4f),clonogenicity (Fig. 5a,b),DNA synthesis (Fig. 5c) and metastasis properties (Fig. 5d). Moreover the inhibition effect of GABARAPL1 siRNA equaled with the inhibition effect of autophagy inhibition drug (HCQ) in the aspect of reversing the biological function of miR-133a-3p on GC cell malignancy. Meanwhile,the inhibitor role of miR-133a-3p mimics on GC malignant behaviors was restored by GABARAPL1 overexpression plasmid (Fig. 4f, 5a,c,d). Besides, the positive role on EMT of miR-133a-3p inhibitors was successfully reversed by GABARAPL1 siRNA and HCQ and the suppressive role on EMT of miR-133a-3p mimics was restored by GABARAPL1 overexpression plasmid, which explained the aforementioned changes on migration and invasion abilities of GC cells in some way (Fig. 5d). Thus, we drew the conclusion that miR-133a-3p could play its tumor suppressor role via targeting GABARAPL1 which blocked the autophagy formation.

**Fig. 5:** Identification of GABARAPL1 as the potential target of miR-133a-3p which is responsible for the autophagy activation and mediating the proliferation and metastasis abilities of GC cells. (**a,b**). Clonogenicity assay demonstrated that the positive role on GC clonogenic formation of miR-133a-3p inhibitors was successfully reversed by GABARAPL1 siRNA and HCQ. (**c**). Edu assay demonstrated that the positive role on GC DNA synthesis of miR-133a-3p inhibitors was successfully reversed by GABARAPL1 siRNA and HCQ, scale bar = 100 μm. (**d**). Transwell assay proved that the positive role on GC metastasis of miR-133a-3p inhibitors was successfully reversed by GABARAPL1 siRNA and HCQ, scale bar = 200 μm. All data are presented as mean ± SEM. *p < 0.05, **p < 0.01, ***p < 0.001

### Glutamine metabolism reveals the specific downstream mechanism of miR-133a-3p mediated autophagy

There have been many reports on various effects of glutamine and its downstream products on tumor proliferation, migration and invasion because of their biological function of supplying carbon and nitrogen atoms for construction of multiple macromolecular precursors. They are reported to play crucial roles in regulating bioenergetics and biosynthesis, gene expression, and anti-oxidative defense [48–50]. Meanwhile, it is generally believed that autophagy could relieve metabolic stress mostly by degrading intracellular components to generate amino acids, fatty acids, sugars, and nucleotides, which are recycled into the TCA cycle and biosynthetic pathways. Glutaminolysis mediated by autophagy favors the tumor cells in the form of downstream glutamate and α-KG through enzymatic processes by glutaminase (GLS) and glutamate dehydrogenase (GDH) respectively. Firstly, we utilized the total candidate genes of miR-133a-3p from miRDB, miRTarBase, miRWalk and TargetScan to perform the Kyoto encyclopedia of genes and genomes (KEGG) analysis on the downstream biological pathway of miR-133a-3p.We found that metabolic pathway alteration is the most important change within the biological pathways mediated by miR-133a-3p (Additional file 1: Figure S1a). Secondly,we utilized the common candidate genes of miR-133a-3p within the aforementioned databases to perform the Gene Ontology (GO) analysis to discover the most potential biological function of miR-133a-3p.We also found that miR-133a-3p has close relationship with macromolecule catabolic process and protein catabolic process (Additional file 1: Figure S1b). Thus, considering the fact that miR-133a-3p could affect autophagy and the close connection between miR-133a-3p and protein catabolism. We tried to investigate whether miR-133a-3p could block glutaminolysis through autophagy and further suppress the malignant behavior of GC cells. Subsequently, we constructed stable clones of LV-miR-NC,LV-miR-133a-3p or LV-miR-133a-3p-IN into MKN-45 and BGC-823 cells (Fig. 6a). Then, the aforementioned GC cells were treated with HCQ, GLS siRNA, BPTES (a GLS inhibition drug) and negative control respectively and were cultured in serum-free RPMI-1640 without glutamine. In the next step, we detected the contents of glutamine, glutamate,α-KG in GC cells by liquid chromatography-mass spectrometry (LC-MS) (Fig. 6b) and the expression level of GLS and GDH by western blot assay (Fig. 7a). As illustrated in the LC-MS results, using HCQ equaled the effect of using GLS siRNA and BPTES in the aspect of glutamine metabolism inhibition, which implied autophagy in GC cells do accelerate the glutaminolysis process. We further confirmed this by means of immunofluorescence with anti-LC3, anti-GLS and anti-GDH (Fig. 7b). We observed the co-activation and co-localization of these three proteins which suggested the strong synergy between autophagy and glutaminolysis. Moreover,all the LV-miR-133a-3p GC cells presented a decreasing trend of autophagy mediated glutaminolysis compared with LV-miR-NC GC cells respectively. The LV-miR-133a-3p-IN GC cell groups demonstrated higher levels of glutaminolysis mediated by autophagy compared with LV-miR-NC GC cells. Moreover, we attempted to figure out whether blocking glutaminolysis could reverse the effects of LV-miR-133a-3p-IN on GC malignant behavior. Edu assay showed that GLS siRNA and BPTES treatment could reverse the positive regulation role of LV-miR-133a-3p-IN on GC cell proliferation (Fig. 7c). Western blot assay and transwell assay demonstrated that blocking glutaminolysis could also prevent the promotion role of LV-miR-133a-3p-IN on EMT (Fig. 7e) and its associated metastasis property of GC cells (Fig. 7d). Based on the results previously discussed, the regulation role of miR-133a-3p on glutaminolysis through autophagy was confirmed.

**Fig. 6:** Glutamine metabolism reveals the specific downstream mechanism of miR-133a-3p mediated autophagy. (**a**). KEGG analysis on the downstream biological pathway of miR-133a-3p. (**b**). We utilized the common candidate genes of miR-133a-3p within the aforementioned databases to perform the Gene Ontology (GO) analysis to discover the most potential biological function of miR-133a-3p. (**c**). Transfection efficiency of LV-miR-NC,LV-miR-133a-3p,LV-miR-133a-3p-IN,miR-133a-3p mimics,miR-133a-3p-IN in MKN-45 and BGC-823 cells. (**d**). LC-MS was chosen to analyze glutaminolysis metabolites and the results showed that using HCQ equaled the effect using GLS siRNA or BPTES in the aspect of glutamine metabolism inhibition. Moreover,miR-133a-3p was observed to block glutaminolysis. All data are presented as mean ± SEM. *p < 0.05, **p < 0.01, ***p < 0.001

**Fig. 7:** Glutamine metabolism reveals the specific downstream mechanism of miR-133a-3p mediated autophagy. (**a**). Western blot assay also showed that using HCQ equals the effect using GLS siRNA and BPTES in the aspect of glutamine metabolism inhibition. Moreover,miR-133a-3p was observed to block glutaminolysis. (**b**). Immunofluorescence with anti-LC3,anti-GLS and anti-GDH showed the co-activation and co-localization of these three proteins which proves the strong synergy between autophagy and glutaminolysis, scale bar = 5 μm. (**c**). Edu assay showed that GLS siRNA and BPTES could reversed the positive regulation of LV-miR-133a-3p-IN on GC cell proliferation, scale bar = 100 μm. (**d**). Transwell assay showed that GLS siRNA and BPTES could reversed the positive regulation of LV-miR-133a-3p-IN on GC cell metastasis, scale bar = 200 μm. (**e**). Western blot assay demonstrated that blocking glutaminolysis could also prevent the promotion role of LV-miR-133a-3p-IN on EMT. All data are presented as mean ± SEM. *p < 0.05, **p < 0.01, ***p < 0.001

### The miR-133a-3p-autophagy-glutaminolysis pathway distributes to a favorable environment for GC cells

Glutamine provides carbon and nitrogen atoms to replenish TCA cycle and redox balance which are responsible for the energy homeostasis and the balance of ROS stress finally favoring GC cells to survive [51, 52]. This inspired us to further validate the effects of the miR-133a-3p-autophagy-glutaminolysis pathway in mediating the survival abilities of GC cells. Firstly,LV-miR-133a-3p,LV-miR-133a-3p-IN and LV-miR-NC GC cells treated with GABARAPL1 siRNA, GLS siRNA and BPTES respectively were subjected to the serum-free RPMI1640 solution. Subsequently, we detected the survival abilities of them by clonogenic survival assay (Fig. 8a) and the relative mitochondrial respiration by oxygen consumption rate (OCR) assay (Fig. 8b) before and after supplementing with glutamine. Obviously, the tumor suppressor role of miR-133a-3p on weakening the survival abilities of GC cells was proved. It was confirmed as well that the autophagy and glutaminolysis inhibition by siRNA and drug could further decrease survival abilities and respiration of LV-miR-133a-3p GC cells. However, it was observed that clonogeic survival abilities and OCR of GC cells were restored to higher levels, when supplemented with glutamine (FI G8a,8b) except the GC cells treated with si GLS. Oxidative phosphorylation produces the largest amount of ATP in humans under normal conditions. Aforementioned results revealed that the oxidative phosphorylation and TCA metabolites (glutamate and α-KG) both decreased in LV-miR-133a-3p cells and were further reduced when blocking either autophagy or glutaminolysis at the same time (Fig. 8b,6d). Therefore, we hypothesized that the miR-133a-3p-autophagy-glutaminolysis pathway plays a crucial role in energy homeostasis and we attempted to detected the ATP generation in the aforementioned groups of GC cells. ATP decreased greatly in LV-miR-133a-3p cells and was even lower in either autophagy or glutaminolysis deficient tumor cells (Fig. 9a). Consistent with the former results, ATP generation was restored when GC cells was supplemented with glutamine except the GC cells treated with si GLS (Fig. 9a). Glutamine metabolism is generally believed to be reprogramed by converting malate to pyruvate for the sake of generating NADPH and further maintaining the cellular redox state under starvation in cancer development. This made us to suspect glutaminolysis via autophagy is necessary for maintaining the redox balance in starvation. To prove our thought, we detected the ROS level in the aforementioned groups of cells (Fig. 9b) under starving condition. Consistent with the aforementioned results, the deficiencies of autophagy and glutaminolysis made the low level of ROS in GC cells caused by LV-miR-133a-3p-IN become even lower. Moreover, the supplementation of glutamine attenuated ROS production which favored the survival condition of GC cells except the GC cells treated with si GLS. We concluded from the aforementioned results that when the core glutaminolysis enzyme GLS was blocked, the rescue effect of glutamine was useless.

**Fig. 8:** The miR-133a-3p-autophagy-glutaminolysis pathway distributes to a favorable environment for GC cells. (**a**). It was confirmed that the autophagy and glutaminolysis inhibition by siRNA and drug could further decrease survival abilities of LV-miR-133a-3p GC cells by clonogenic survival assay. (**b**). It was confirmed as well that the autophagy and glutaminolysis inhibition by siRNA and drug could further decrease mitochondrial respiration of LV-miR-133a-3p GC cells by oxygen consumption rate (OCR) assay. All data are presented as mean ± SEM. *p < 0.05, **p < 0.01, ***p < 0.001

**Fig. 9:** The miR-133a-3p-autophagy-glutaminolysis pathway distributes to a favorable environment for GC cells. (**a**). ATP decreased greatly in LV-miR-133a-3p cells and was even lower in either autophagy or glutaminolysis deficient tumor cells, scale bar = 100 μm. (**b**). The deficiencies of autophagy and glutaminolysis made the low level of ROS in GC cells caused by LV-miR-133a-3p-IN become even lower. (**c**). Working pattern of miR-133a-3p regulating GC malignant behavior via autophagy mediated glutaminolysis. All data are presented as mean ± SEM. *p < 0.05, **p < 0.01, ***p < 0.001

We thereby proved that the process of miR-133a-3p mediating glutaminolysis via autophagy could support the survival abilities of GC cells through energy homeostasis and redox balance and the working pattern was shown in Fig. 9c.

### miR-133a-3p blocks GC growth and metastasis better with the combination of autophagy and glutaminolysis inhibitors in vivo

It is publicly recognized that the patient-derived xenograft (PDX) mice model was applied to study human cancer cells under controlled conditions and can be especially useful for preclinical studies of therapeutics [53]. Thus, we utilized this model to determine the therapeutic effects of using LV-miR-133a-3p alone or combination of HCQ and BPTES on GC growth. We adopted intratumoral injection of recombinant LV-miR-133a-3p,LV-miR-133a-3p-IN,LV-miR-NC,LV-miR-133a-3p plus HCQ and BPTES on four groups of PDX mice respectively (Fig. 10a). Next, we clinically characterized the donor patients and histopathologically analyzed the xenografted tumors (Fig. 10b,c).MiR-133a-3p remarkably decreased in these 3 GC clinical specimens when compared to the adjacent normal tissues (Fig. 10b). Moreover, we observed lower weight and volume of the xenografted tumors under LV-miR-133a-3p treatment compared with the LV-NC group (Fig. 10d), and the tumor growth was further blocked under the combination of drug treated groups. Oppositely, the tumor growth was accelerated under LV-miR-133a-3p-IN treatment. Furthermore, qRT-PCR was performed in PDX tumors, and we found increased and persistent level of miR-133a-3p in LV-miR-133a-3p treated groups compared with the NC group and the lower level of miR-133a-3p in LV-133a-3p-IN groups. We even found a much lower level of miR-133a-3p in the drug-combined groups (Fig. 10e). Afterwards we determined the expression levels of LC3, GLS and GDH in the four groups of PDX tumors by immunohistochemistry (Fig. 10f) and western blot (Fig. 10I). We observed the increased LC3, GLS and GDH levels in the miR-133a-3p-treated tumor cells. On the contrary, weakened autophagy and glutaminolysis were observed in LV-miR-133a-3p-treated group. Moreover, we observed even lower autophagy and glutaminolysis in drug treated groups. We detected higher GABARAPL1 and ATG13 expressions when miR-133a-3p-IN was engaged and discovered ever much higher expressions in drug treated groups compared with the other groups (Fig. 10I). In addition, we attempted to detect the regulation role of miR-133a-3p on distant metastasis via tail vein injection into BALB/c Nude mice with LV-miR-133a-3p,LV-NC and LV-miR-133a-3p IN GC cells. We observed the mostly lung metastasis and few peritoneal metastasis by detecting the luciferase intensities every week until four weeks. According to the luciferase intensities detected in thoracic cavity, we found that miR-133a-3p could block the lung metastasis (Fig. 10g). Next, we harvested the lung tissues for H&E staining (Fig. 10h) to show their pathological characters. The results were consistent with the luciferase intensities detection in three groups of mice that LV-miR-133a-3p IN GC cells had the biggest promotor role on distant organ metastasis. Considering the role of miR-133a-3p on EMT verified in vitro, we again demonstrated the suppressor role of miR-133a-3p on metastasis via EMT mechanism in the aforementioned PDX tumor tissues in vivo (Fig. 10I). From the previously discussed results, the conclusion can be arrived at that the injection of LV-miR-133a-3p could successfully reduce the growth of PDX tumors by interfering glutaminolysis via inhibition of autophagy and block the distant organ metastasis of GC via inhibiting EMT mechanism. Furthermore, the combination of LV-miR-133a-3p and autophagy inhibitor HCQ and glutaminolysis could bring about a better therapeutic outcome on limiting tumor growth.

**Fig. 10:** miR-133a-3p blocks GC growth and metastasis better with the combination of autophagy and glutaminolysis inhibitors in vivo. (**a**). Procedures of establishing PDX model. (**b**). Clinical characteristics of the donor patients. (c). H&E staining of the donor patients’ tissues, scale bar = 100 μm. (**d**). Lower weight and volume of the xenografted tumors could be observed under LV-miR-133a-3p treatment compared with the LV-NC and LV-miR-133a-3p-IN groups and the tumor growth was further inhibited under drug-combination groups. (**e**). We found increased and persistent level of miR-133a-3p in LV-miR-133a-3p treated groups compared with the LV-NC group and a much higher level of miR-133a-3p in the drug-combination groups. (**f**). We determined the LC3,GLS and GDH levels in the different groups of PDX tumors by immunohistochemistry, scale bar = 100 μm. (**g**). We determined the role of miR-133a-3p on metastasis in vivo by tail vein injection LV-miR-133a-3p.LV-NC,LV-miR-133a-3p IN GC cells and we than measured the luciferase intensities each week. (**h**). We took H&E staining to show the lung metastasis foci. (**i**). The expression level of LC3,P62,GLS,GDH,GABARAPL1, ATG13 and EMT markers in PDX tumors was determined by western blot. All data are presented as mean ± SEM. *p < 0.05, **p < 0.01, ***p < 0.001

## Discussion

Glutaminolysis has now been recognized as an important hallmark of tumor metabolism. Researchers have focused their studies on glutamine rather than glucose in the terms of tumor cell metabolism over the past few years. Biosynthesis, bioenergetics and ROS homeostasis are three major ways that glutaminolysis takes to promote tumor cell proliferation, migration and invasion. Glutaminolysis could replenish the TCA cycle by providing α-KG to produce both adequate ATP and substrates for biosynthesis. In addition, glutaminolysis also helps synthesis of nucleotides by donating nitrogen to purines and pyrimidines and synthesis of certain nonessential amino acids. In this case, glutamine acts as a carbon and nitrogen donor which is necessary for survival of tumor cells. Concerning the tumor promotor role of glutaminolysis, FDA approved many kinds of glutaminolysis inhibitors to go into clinical trials [54–56]. Apart from the metabolism alterations in tumor cells, it is also discovered that tumor can be usually identified as elevated autophagy to buffer the nutrients limitations. Many researchers reported the higher autophagy level within GC tumor were correlated with the shorter survival of GC patient. According to our investigation, the basal autophagy level of gastric cancer cells is higher than normal stomach epithelial cells. In the past few years, connections between autophagy and metabolism have been discovered, but the deeper regulation mechanisms of them on GC development have not been understood comprehensively. According to our study, autophagy involved in the glutaminolysis provides necessary glutamine metabolism products which eventually rescue GC cell survival. Inhibition of autophagy almost phenocopied the effect of directly blocking glutaminolysis on suppressing tumor deveolopment. Additionally, it was reported that the positive correlation between autophagy and EMT mediated metastasis. Considering the promotion effect of autophagy on glutaminolysis and EMT, we tried to found a method targeting autophagy to block GC growth and metastasis.

MiRNA is a kind of noncoding RNA that can post-transcriptionally regulate its targeting gene expression. Many researchers have reported that miR-133a-3p could function in prostate cancer, gastric cancer and bladder cancer as a tumor suppressor. As several researchers reported that miR-133a-3p is crucial in a series pathological and biological processes by regulating different genes, such as Her-2, EGFR, Snai1, and Evi1.However, the investigation about the exact role of miR-133a-3p on regulating autophagy, glutaminolysis and EMT have not been clarified. As we observed, miR-133a-3p blocked the activation of autophagy and glutaminolysis in GC cells, which prompts our further exploration on the deeper interaction between autophagy and glutaminolysis under the mediation of miR-133a-3p.The advancement of our reports is the utilization of certain models to investigate the biological role of miR-133a-3p.We combined organoid model and PDX model to verify the tumor suppressor role of miR-133a-3p both in vitro and in vivo. Organoid model consists of several types of GC cells that grow with three dimensional structures and phenocopies the micro-environment of primary GC tissues. PDX model is also retained the vivo micro environment and can more easily forecast the therapeutic efficiency. Therefore, these two models reduce the possibility of GC cells from intentionally or unintentionally population selecting. We used organoid model and PDX model to verify the inhibition role of miR-133a-3p role on autophagy mediated glutaminolysis. Additionally, we determined the suppress role of miR-133a-3p on EMT in GC cells and detected the distant organ metastasis via scan on BALB/c nude mice which were injected luciferase-labeled lentivirus.

Over the past few years, researchers have reported many miRNAs could interact the glutaminolysis including miR-204,miR-137,miR-192 and miR-23a/b [57–59]. According to our study, it is found that miR-133a-3p could block the activation of glutaminolysis by reducing the expression level of core enzymes including GLS and GDH, but not directly targeting them at the posttranscriptional level. Besides, we found that miR-133a-3p could mediate autophagy in GC cells by directly regulating ATGs, including GABARAPL1 and ATG13.It is reported that GABARAP subfamily proteins can, more efficiently than LC3–2, serve as scaffolding proteins by recruiting ULK1 and beclin-1 (complex) to the site of autophagosome nucleation and directly participant autophagy. ATG13 is an autophagy initiator which are contained in ATG13-ULK1-RB1CC1 complex. Its regulation on ULK1 activity plays an important role in mediating the kinase activity of mTORC1 and cell proliferation. We found that LV-miR-133a-3p GC cells could block the expression of these two targets at both mRNA and protein level further demonstrating that miR-133a-3p is an autophagy regulator.

## Conclusions

To sum up, miR-133a-3p could target autophagy and further affect both glutaminolysis and EMT which made itself a tumor suppressor. We found that the overexpression of miR-133a-3p could block the proliferation, migration and invasion abilities of GC cells. Organoid models were taken to prove the autophagy alteration inhibited by miR-133a-3p and the tumor suppressor role of miR-133a-3p.In addition, we discovered the decreased glutaminolysis level under the inhibition of autophagy by chemical inhibitors HCQ or miR-133a-3p overexpression. Finally, the PDX model demonstrated that miR-133a-3p overexpression could block the autophagy mediated glutaminolysis in vivo.LV-miR-133a-3p could also successfully decrease the tumor weight and volume and proved itself as a tumor suppressor. Moreover,the combination use of HCQ and BPTES could further increase the theraputic effect of LV-miR-133a-3p.Besides, the results of luciferase scan on mice which were received tail vein injection of luciferase-labeled GC cells proved the inhibition role of miR-133a-3p on distant organ metastasis. To summarize, overexpression of miR-133a-3p might be a promising therapeutic strategy against GC development.

## Additional file

Additional file 1: **Figure S1.** Bioinfomatic analysis of downstream genes of miR-133a-3p. **A.** we utilized the total candidate genes of miR-133a-3p from miRDB, miRTarBase, miRWalk and TargetScan to perform the Kyoto encyclopedia of genes and genomes (KEGG) analysis on the downstream biological pathway of miR-133a-3p. **B.** We utilized the common candidate genes of miR-133a-3p within the aforementioned databasesto perform the Gene Ontology (GO) analysis to discover the most potential biological function of miR-133a-3p. (TIF 2230 kb)

## List of abbreviations

GC: Gastric cancer.
HCQ: Hydroxychloroquine.
miR-133a-3p: microRNA-133a-3p.
EMT: Epithelial-mesenchymal transition.
PDX: Patient-derived xenograft.
GABARAPL1: GABARAP-like protein 1.
3′-UTR: 3′-untranslated regions.
GAU: The 3’-UTR (3′-untranslated region) of GABARAPL1.
GAU-WT: The wide type of putative miR-133a-3p binding sequence.
GAU-MT: The mutant type of putative miR-133a-3p binding sequence.
qRT-PCR: Quantitative real-time PCR.

## References

[1] Torre LA (2015). Global cancer statistics, 2012. CA Cancer J Clin.

[2] Zhou H (2016). Autophagy regulation and its role in gastric cancer and colorectal cancer. Cancer Biomark.

[3] Isobe T (2013). Clinicopathological significance of hypoxia-inducible factor-1 alpha (HIF-1alpha) expression in gastric cancer. Int J Clin Oncol.

[4] Yuan LW, Yamashita H, Seto Y (2016). Glucose metabolism in gastric cancer: the cutting-edge. World J Gastroenterol.

[5] Parzych KR, Klionsky DJ (2014). An overview of autophagy: morphology, mechanism, and regulation. Antioxid Redox Signal.

[6] Maes H (2013). Autophagy: shaping the tumor microenvironment and therapeutic response. Trends Mol Med.

[7] White E, Mehnert JM, Chan CS (2015). Autophagy, metabolism, and Cancer. Clin Cancer Res.

[8] Xu XD (2015). Warburg effect or reverse Warburg effect? A review of cancer metabolism. Oncol Res Treat.

[9] Liberti MV, Locasale JW (2016). The Warburg effect: how does it benefit Cancer cells?. Trends Biochem Sci.

[10] Chen JQ, Russo J (2012). Dysregulation of glucose transport, glycolysis, TCA cycle and glutaminolysis by oncogenes and tumor suppressors in cancer cells. Biochim Biophys Acta.

[11] Jin L, Alesi GN, Kang S (2016). Glutaminolysis as a target for cancer therapy. Oncogene.

[12] Yang C (2014). Glutamine oxidation maintains the TCA cycle and cell survival during impaired mitochondrial pyruvate transport. Mol Cell.

[13] Yang L (2014). Metabolic shifts toward glutamine regulate tumor growth, invasion and bioenergetics in ovarian cancer. Mol Syst Biol.

[14] Wise DR, Thompson CB (2010). Glutamine addiction: a new therapeutic target in cancer. Trends Biochem Sci.

[15] Gonzalez CD (2014). Autophagy, Warburg, and Warburg reverse effects in human cancer. Biomed Res Int.

[16] Villar VH (2015). Glutaminolysis and autophagy in cancer. Autophagy.

[17] Strohecker AM (2013). Autophagy sustains mitochondrial glutamine metabolism and growth of BrafV600E-driven lung tumors. Cancer Discov.

[18] Lu WH (2014). Autophagy functions on EMT in gastrulation of avian embryo. Cell Cycle.

[19] Pang M (2016). Autophagy links beta-catenin and Smad signaling to promote epithelial-mesenchymal transition via upregulation of integrin linked kinase. Int J Biochem Cell Biol.

[20] Hardy SD (2017). Regulation of epithelial-mesenchymal transition and metastasis by TGF-beta, P-bodies, and autophagy. Oncotarget.

[21] Wang RC (2012). Akt-mediated regulation of autophagy and tumorigenesis through Beclin 1 phosphorylation. Science.

[22] Dunlop EA, Tee AR (2014). mTOR and autophagy: a dynamic relationship governed by nutrients and energy. Semin Cell Dev Biol.

[23] Zong H (2014). Inhibition of mTOR pathway attenuates migration and invasion of gallbladder cancer via EMT inhibition. Mol Biol Rep.

[24] Xu W, Yang Z, Lu N (2015). A new role for the PI3K/Akt signaling pathway in the epithelial-mesenchymal transition. Cell Adhes Migr.

[25] Tanida I (2011). Autophagosome formation and molecular mechanism of autophagy. Antioxid Redox Signal.

[26] John CD (2016). MiR-26b inhibits autophagy by targeting ULK2 in prostate cancer cells. Biochem Biophys Res Commun.

[27] Sun KT (2015). MicroRNA-20a regulates autophagy related protein-ATG16L1 in hypoxia-induced osteoclast differentiation. Bone.

[28] Guo X (2015). MiR224-3p inhibits hypoxia-induced autophagy by targeting autophagy-related genes in human glioblastoma cells. Oncotarget.

[29] Shin VY, Chu KM (2014). MiRNA as potential biomarkers and therapeutic targets for gastric cancer. World J Gastroenterol.

[30] Huang YK, Yu JC (2015). Circulating microRNAs and long non-coding RNAs in gastric cancer diagnosis: an update and review. World J Gastroenterol.

[31] Acunzo M (2015). MicroRNA and cancer--a brief overview. Adv Biol Regul.

[32] Tao J (2012). microRNA-133 inhibits cell proliferation, migration and invasion in prostate cancer cells by targeting the epidermal growth factor receptor. Oncol Rep.

[33] Zhang XT (2015). Impairment of growth of gastric carcinoma by miR-133-mediated Her-2 inhibition. Tumour Biol.

[34] Zhou Y (2013). MicroRNA-133 inhibits cell proliferation, migration and invasion by targeting epidermal growth factor receptor and its downstream effector proteins in bladder cancer. Scand J Urol.

[35] Su Z (2015). MicroRNAs in apoptosis, autophagy and necroptosis. Oncotarget.

[36] Yu X (2015). MiR-214 increases the sensitivity of breast cancer cells to tamoxifen and fulvestrant through inhibition of autophagy. Mol Cancer.

[37] Atherton DS (2016). Factors affecting the use of human tissues in biomedical research: implications in the design and operation of a biorepository. Methods Mol Biol.

[38] Marano L (2015). Comparison of the 6th and 7th editions of the AJCC/UICC TNM staging system for gastric cancer focusing on the "N" parameter-related survival: the monoinstitutional NodUs Italian study. World J Surg Oncol.

[39] Mahe MM (2013). Establishment of gastrointestinal epithelial organoids. Curr Protoc Mouse Biol.

[40] Avila-Ospina L (2014). Autophagy, plant senescence, and nutrient recycling. J Exp Bot.

[41] Filomeni G, De Zio D, Cecconi F (2015). Oxidative stress and autophagy: the clash between damage and metabolic needs. Cell Death Differ.

[42] Jiang X, Overholtzer M, Thompson CB (2015). Autophagy in cellular metabolism and cancer. J Clin Invest.

[43] Mathew R, White E (2011). Autophagy, stress, and cancer metabolism: what doesn't kill you makes you stronger. Cold Spring Harb Symp Quant Biol.

[44] Su Z (2017). Autophagy inhibition impairs the epithelial-mesenchymal transition and enhances cisplatin sensitivity in nasopharyngeal carcinoma. Oncol Lett.

[45] Luo D (2018). Mesenchymal stem cells promote cell invasion and migration and autophagy-induced epithelial-mesenchymal transition in A549 lung adenocarcinoma cells. Cell Biochem Funct.

[46] Hervouet E (2015). The autophagy GABARAPL1 gene is epigenetically regulated in breast cancer models. BMC Cancer.

[47] Lebovitz CB (2015). Cross-cancer profiling of molecular alterations within the human autophagy interaction network. Autophagy.

[48] Li C (2016). Metabolic reprogramming in cancer cells: glycolysis, glutaminolysis, and Bcl-2 proteins as novel therapeutic targets for cancer. World J Surg Oncol.

[49] Ge Y (2015). MiRNA-192 [corrected] and miRNA-204 directly suppress lncRNA HOTTIP and interrupt GLS1-mediated Glutaminolysis in hepatocellular carcinoma. PLoS Genet.

[50] Friday E (2011). Glutaminolysis and glycolysis regulation by troglitazone in breast cancer cells: relationship to mitochondrial membrane potential. J Cell Physiol.

[51] Alberghina L, Gaglio D (2014). Redox control of glutamine utilization in cancer. Cell Death Dis.

[52] Weinberg F (2010). Mitochondrial metabolism and ROS generation are essential for Kras-mediated tumorigenicity. Proc Natl Acad Sci U S A.

[53] Aparicio S, Hidalgo M, Kung AL (2015). Examining the utility of patient-derived xenograft mouse models. Nat Rev Cancer.

[54] Jacque N (2015). Targeting glutaminolysis has antileukemic activity in acute myeloid leukemia and synergizes with BCL-2 inhibition. Blood.

[55] Cervantes-Madrid D, Duenas-Gonzalez A (2015). Antitumor effects of a drug combination targeting glycolysis, glutaminolysis and de novo synthesis of fatty acids. Oncol Rep.

[56] Guo L (2016). Blockage of glutaminolysis enhances the sensitivity of ovarian cancer cells to PI3K/mTOR inhibition involvement of STAT3 signaling. Tumour Biol.

[57] Correction: fMiRNA-192 and miRNA-204 Directly Suppress lncRNA HOTTIP and Interrupt GLS1-Mediated Glutaminolysis in Hepatocellular Carcinoma. PLoS Genet. 2016;12(1):e1005825.10.1371/journal.pgen.1005825PMC472663426807954

[58] Luo M, et al. miR-137 regulates ferroptosis by targeting glutamine transporter SLC1A5 in melanoma. Cell Death Differ. 2018.10.1038/s41418-017-0053-8PMC611331929348676

[59] Kou Y, Zheng WT, Zhang YR (2016). Inhibition of miR-23 protects myocardial function from ischemia-reperfusion injury through restoration of glutamine metabolism. Eur Rev Med Pharmacol Sci.

